# Anti-Oxidative Defences Are Modulated Differentially in Three Freshwater Teleosts in Response to Ammonia-Induced Oxidative Stress

**DOI:** 10.1371/journal.pone.0095319

**Published:** 2014-04-16

**Authors:** Amit Kumar Sinha, Hamada AbdElgawad, Terri Giblen, Gaurav Zinta, Michelle De Rop, Han Asard, Ronny Blust, Gudrun De Boeck

**Affiliations:** 1 Systemic Physiological and Ecotoxicological Research, Department of Biology, University of Antwerp, Antwerp, Belgium; 2 Molecular Plant Physiology and Biotechnology group, Department of Biology, University of Antwerp, Antwerp, Belgium; Institut National de la Recherche Agronomique (INRA), France

## Abstract

Oxidative stress and the antioxidant response induced by high environmental ammonia (HEA) were investigated in the liver and gills of three freshwater teleosts differing in their sensitivities to ammonia. The highly ammonia-sensitive salmonid *Oncorhynchus mykiss* (rainbow trout), the less ammonia sensitive cyprinid *Cyprinus carpio* (common carp) and the highly ammonia-resistant cyprinid *Carassius auratus* (goldfish) were exposed to 1 mM ammonia (as NH_4_HCO_3_) for 0 h (control), 3 h, 12 h, 24 h, 48 h, 84 h and 180 h. Results show that HEA exposure increased ammonia accumulation significantly in the liver of all the three fish species from 24 h–48 h onwards which was associated with an increment in oxidative stress, evidenced by elevation of xanthine oxidase activity and levels of hydrogen peroxide (H_2_O_2_) and malondialdehyde (MDA). Unlike in trout, H_2_O_2_ and MDA accumulation in carp and goldfish liver was restored to control levels (84 h–180 h); which was accompanied by a concomitant increase in superoxide dismutase (SOD), catalase (CAT), ascorbate peroxidase activity and reduced ascorbate content. Many of these defence parameters remained unaffected in trout liver, while components of the glutathione redox cycle (reduced glutathione, glutathione peroxidase and glutathione reductase) enhanced to a greater extent. The present findings suggest that trout rely mainly on glutathione dependent defensive mechanism while carp utilize SOD, CAT and ascorbate as anti-oxidative sentinels. Hepatic cells of goldfish appear to utilize each of these protective systems, and showed more effective anti-oxidative compensatory responses towards HEA than carp, while trout were least effective. The present work also indicates that HEA exposure resulted in a relatively mild oxidative stress in the gills of all three species. This probably explains the almost complete lack of anti-oxidative responses in branchial tissue. This research suggests that oxidative stress, as well as the antioxidant potential clearly differ between salmonid and cyprinid species.

## Introduction

In confined waters and in aquaculture systems, a possible accumulation of metabolic waste products of fish, including ammonia can rapidly rise to unsafe levels. Moreover, ammonia also enters the water bodies from sources such as sewage effluents, industrial wastes, agricultural run-off and decomposition of biological wastes [1]. Waterborne ammonia can exist in two forms, the unionized ammonia (NH_3_) and the ionized form (NH_4_^+^), and the sum of NH_3_ and NH_4_^+^ comprises the total ammonia concentration. Throughout this paper, the term ‘ammonia’ is used to refer to total ammonia. The build-up of high environmental ammonia (HEA) may become a serious threat for aquatic animals, including fish. At HEA, ammonia excretion in fish is hindered and/or net uptake of ammonia from the environment occurs. This leads to a situation where fish are confronted simultaneously with accumulation of endogenous ammonia and uptake of exogenous ammonia. As a result, blood and tissue ammonia levels increase and fish experience both acute and chronic toxic effects [2]–[4]. Notable pathologies include decreased growth rates [2], [3], [5]–[7], alterations in energy metabolism [8], disruption of ionic balance [9]–[11], alterations in hormone regulation [2], [12], increased vulnerability to disease and histopathological changes in gill epithelia [11], cause neurotoxicity such as astrocyte swelling [13], [14], glutamate excitotoxicity particularly over-activation of *N*-methyl-D-aspartate type glutamate (NMDA) receptors [15]–[16], and the generation of reactive oxygen species(ROS) [17]. At high levels, HEA even induces hyperexcitability, coma, convulsions and death. Many teleosts have evolved a number of different strategies to defend against ammonia toxicity [18]–[20]. These include- conversion of accumulated ammonia to glutamine and other free amino acids, reduction in ammonia production by suppressing amino acid catabolism and/or partial amino acid catabolism, detoxification of ammonia to the less toxic urea possibly through the ornithine urea cycle, and augmentation of ammonia excretion against the gradient by up-regulation of ‘Na^+/^NH_4_^+^ exchange complex or metabolon’ involving the Rh glycoproteins [21]. Numerous studies on different fish species concerning acute and chronic ammonia toxicity already exist [2], [3], [12], [22]–[29], however ammonia mediated oxidative toxicity, and the response of anti-oxidative defence mechanisms in fish are not yet fully understood.

There is growing evidence that ammonia exposure can lead to oxidative stress in fish species. HEA induced oxidative aberrations were reported in brain and gills of mudskipper, *Boleophthalmus boddarti* [30], liver and muscle of Nile tilapia, *Oreochromis niloticus* [31] and in bighead carp larvae, *Hypophthalmythys nobilis* [32]. Oxidative stress is caused by the production of ROS such as superoxide (O_2_^• −^), hydrogen peroxide (H_2_O_2_), peroxyl (ROO^•^), and hydroxyl radicals (^•^OH). These are generated as by-products of oxidative metabolism, and are responsible for the build-up of oxidized and damaged lipids and proteins in the cell and the cellular compartments [33]. These can lead to loss of cellular or organelle membrane integrity, inactivation of enzymes, metabolic dysfunction, pathological injury and cell death.

Oxidative stress is the consequence of an imbalance between oxidative and reductive processes in the cell. Oxidative stress is induced when the physiological antioxidant defence system can no longer counteract the elevated ROS levels [34], [35], or as a result of the cellular incompetency to repair oxidative damage [36]. These circumstances are manifested by an increase in lipid hydroperoxides, which are estimated through malondialdehyde (MDA) quantification. Similar to other vertebrates, teleosts have evolved a wide array of antioxidant defence systems to protect themselves from deleterious effect of ROS [37]–[39]. These comprise low molecular weight anti-oxidants such as reduced glutathione (GSH) and ascorbate (ASC), and high-molecular weight defences include enzymes such as superoxide dismutase (SOD), catalase (CAT), glutathione peroxidase (GPX), glutathione reductase (GR), glutathione-s-transferase (GST) and ascorbate peroxidase (APX) [40]–[43]. These enzymatic and non-enzymatic constituents scavenge free radical elements and protect the cell against oxidative damage [44], [45]. The induction in antioxidants can vary considerably between fish species depending on their resilience to the contaminants causing oxidative damage [46], [47]. Therefore, we postulated that oxidative stress and countervailing response of enzymatic and non-enzymatic antioxidants vary among fish species with different tolerance limits to ammonia toxicity. Understanding these differences might help to identify underlying mechanisms involved in ammonia sensitivity. Therefore, the focus of the present comparative study was to elucidate oxidative stress and anti-oxidative defence responses in vital organs such as gills and liver of three commercially important freshwater fish differing in their sensitivities to ammonia: a sensitive salmonid, the rainbow trout *Oncorhynchus mykiss*, a less sensitive cyprinid, the common carp, *Cyprinus carpio*, and a very resistant cyprinid, the goldfish, *Carassius auratus*, when exposed acutely (3 h) and chronically (up to 180 h) to high environmental ammonia (1 mM; pH 7.9). The reported ammonia 96 h LC_50_ values (expressed as total ammonia) for goldfish, common carp and rainbow trout juveniles are ∼4.2 mM (pH 8.0), 2.6 mM (pH 7.5–7.8) and 1.7 mM (pH 8.0) respectively [48]–[52].

In general, fish gills are directly exposed to exogenous ammonia during HEA exposure. Exogenous ammonia must permeate through the branchial epithelia before being transported through the blood to the liver and other organs. As a dynamic respiratory and osmo-regulatory organ, fish gills are expected to possess a high capacity to produce ROS. However, to date, very limited information is available on whether fish gills would be confronted with oxidative stress during HEA exposure. In general, livers of vertebrates are the main organs of biotransformation, and therefore, they are the preferred organ for monitoring the effects of chemical pollution. Similar to gills, there is little information on whether ammonia would induce oxidative stress in fish liver. Usually, ammonia intoxication (in mammals) is mediated by activation of NMDA receptors, excessive activation leads to oxidative stress [17], [53]. The examination of gills and liver tissues that lack NMDA receptors will therefore also assist to verify alternative routes by which ammonia can induce oxidative stress in non-brain tissue.

In brief, the purpose of this study was two-fold. First, to investigate the level of oxidative damage in these three fish species under ammonia threat by quantifying the indices of oxidative stress (e.g. H_2_O_2_, MDA and XO). Second, to understand the anti-oxidant defence system in response to HEA by comprehensive analysis of antioxidant molecules (GSH and ASC) and enzymes (SOD, CAT, APX, GPX, GR and GST). These findings will offer a better insight into the differences in antioxidant defence mechanisms in these fish species and whether they contribute to the differences in the sensitivity to HEA.

Overall, the results indicate that these fish species show differential anti-oxidative compensatory responses toward HEA. Defensive strategies associated with anti-oxidation system are more effective in goldfish in dealing with the ammonia challenge followed by carp and trout. This perhaps explains in part the high resistance of goldfish towards HEA.

## Materials and Methods

### Experimental system and animals

Rainbow trout, *Oncorhynchus mykiss*, were obtained from a fish farm - Pisciculture Collette, Bonlez, Belgium; goldfish, *Carassius auratus*, were obtained from Aqua Hobby, Heist op den Berg, Belgium; common carp, *Cyprinus carpio*, were obtained from the fish hatchery at Wageningen University, The Netherlands. Fish were kept at the University of Antwerp in aquaria (200 L) for at least a month before the exposure started. Thereafter, a total of 96 goldfish, 96 common carp and 96 rainbow trout were distributed species wise into four 200 L tanks (n = 24 per tank). Average mass (mean ± standard deviation) of rainbow trout was 15±2 g, of common carp 18±3 g, and of goldfish 17±3 g. Each of the tanks was equipped with a recirculating water supply in a climate chamber where temperature was adjusted at 17±1°C and photoperiod was 12 h light and 12 h dark. Temperature can affect ammonia toxicity to aquatic species; therefore, the temperature consistency (17±1°C) was monitored every day. Water quality was ensured through an additional bio-filter containing wadding, activated charcoal and lava stones. Water parameters were: pH 7.4±0.2, dissolved oxygen 6.9–7.4 mg/L, ammonia 0.006–0.009 mM, nitrite 0.0015–0.0021 mM, nitrate 0.015–0.042 mM, Ca^2+^ 0.8–1.0 mM, Mg^2+^ 0.19–0.21 mM, Na^+^ 1.2–1.4 mM, K^+^ 0.09–0.10 mM, Cl^−^ 0.9–1.2 mM, titratable alkalinity 1.6–1.8 mM and hardness 226 mg CaCO_3_/L. Fish were acclimated to the above mentioned constant temperature and photoperiod for 2 weeks prior to the experiment and were fed ad libitum once a day with either commercial pellets (‘Hikari Staple’, Kyorin Food Ind. Ltd., Japan) for common carp and goldfish, or ‘Trouvit’ (Trouw Nutrition, Fontaine-les-Vervins, France) for rainbow trout. Feeding was suspended 2 days before experimentation, which provided sufficient time for the gut to be emptied and to stabilize the endogenous fraction of nitrogenous waste excretion. All animal experiments were approved by the local ethics committee, University of Antwerp (Permit Number: LA1100134), and conducted according to the guidelines of the Federation of European Laboratory Animal Science Associations.

### Exposure and sampling intervals

The experimental set up consisted of exposing the goldfish, carp and trout to 1 mM ammonia for a period of 3 h, 12 h, 24 h, 48 h, 84 h and 180 h. This concentration represents 24%, 38% and 59% of the 96 h LC_50_ values for goldfish, carp and trout, respectively (see Introduction for references). The exposure was conducted in 8 L glass aquaria (water volume set to 6 L). Control groups (no HEA) were setup in parallel to 12 h, 84 h and 180 h exposure groups. The experimental aquaria were shielded with black plastic to minimize visual disturbance and fitted with individual air-stones.

Fish (n = 2) were placed in an individual glass aquaria the evening before an experiment and left overnight to settle with continuous aeration. The experimental protocols consisted of exposing 8 fish (in 4 aquaria) per experiment to HEA. Each exposure aquaria was spiked with the required amount of an NH_4_HCO_3_ stock solution (Sigma, Germany). A constant concentration of 1.08±0.06 mM of ammonia was maintained throughout the experiment. Exposure ammonia concentrations were measured (using the salicylate-hypochlorite method [54]) 6 h after the onset of treatment and the concentration of ammonia in the aquaria was maintained by adding calculated amount of the NH_4_HCO_3_ solution. Moreover, to avoid the microbial breakdown of test chemical and build-up of other waste products, 60–80% of the water was discarded after each 2 days and replaced with fresh water containing the respective amount of ammonia. Water pH was monitored throughout the experimental period and was maintained constantly at 7.8–8.0 via the drop-wise addition of 0.1 mol/L HCL and/or KOH to the water using a polyethylene, disposable transfer pipette. pH was determined using a pH electrode (Hamilton Bonaduz AG, Metrohm) connected to the pH meter.

### Sampling procedure and sample analysis

For sampling, fish were removed from aquaria (n = 8), anesthetized using an overdose of neutralized MS222 (pH 8.0, ethyl 3-aminobenzoate methane-sulfonic acid, 1 g/L, Acros Organics, Geel, Belgium). Fish were dissected on ice; gill and liver were removed, snap frozen in liquid nitrogen, and stored at −80°C for determination of ammonia content, oxidative stress parameters, antioxidant molecules and enzymes. Ammonia content in tissue was determined according to Wright et al. [55] using an enzymatic kit (R-Biopharm AG, Darmstadt, Germany).

### Indices of oxidative stress

#### Quantification of H_2_O_2_

50 mg of each liver and gill tissues were homogenized in 50 mM phosphate buffer (pH 6.5) using MagNALyser (Roche, Vilvoorde, Belgium). H_2_O_2_ concentration in homogenate was measured by the FOX1 method [56], based on the peroxide-mediated oxidation of Fe^2+^, followed by reaction of Fe^3+^ with xylenol orange. Absorbance of the Fe^3+^-xylenol orange complex was measured at 560 nm. Standard curve was obtained by diluting 30% H_2_O_2_.

#### Quantification of lipid peroxidation (MDA measurement)

Malonyldialdehyde (MDA) content, an end product of lipid peroxidation was assayed according to the method of Hodges et al. [57]. 50 mg of tissues was homogenized in 1 mL of 80% ethanol and reacted with thiobarbituric acid to produce pinkish red chromogen thiobarbituric acid-malondialdehyde (TBA-MDA). Absorbance at 440, 532 and 600 nm was measured using in a microplate reader.

### Enzyme assay

Superoxide dismutase (SOD), peroxidase (POX), catalase (CAT), glutathione peroxidadase (GPX), ascorbate peroxidase (APX), glutathione reductase (GR), glutathione-s- transferase (GST) and xanthine oxidase (XO) were determined from the homogenate prepared in 1 mL of 50 mM potassium phosphate buffer (pH 7.0) containing 10% polyvinyl pyrrolidone (PVP), 0.25% Triton X-100, 0.001 M polymethyl sulfonyl fluoride (PMSF) and 0.001 M ascorbate using MagNALyser. All activity measurements were scaled down for semi-high throughput using a micro-plate reader (Synergy Mx, Biotek Instruments Inc., Vermont, USA), and optimized to obtain linear time and protein-concentration dependence. SOD activity was determined according to Dhindsa et al. [58] by measuring the inhibition of nitroblue tetrazolium (NBT) reduction at 560 nm. SOD activity was quantified by using a standard curve using known units of purified SOD enzyme under identical conditions against the % of NBT reduction. CAT activity was assayed according to the procedure of Aebi [59] by monitoring the rate of decomposition of H_2_O_2_ at 240 nm. GPX activity was assayed according to Drotar et al. [60] by measuring the decrease in NADPH absorbance measured at 340 nm and calculated from the 6.22 mM^−1^ cm^−1^ extinction coefficient. APX and GR activities were measured by the method of Murshed et al. [61]. APX activity was determined by measuring the decrease in reaction rate at 290 nm and calculated from the 2.8 mM^−1^ cm^−1^ extinction coefficient. GR activity was determined by measuring the decrease in reaction rate at A_340_ and calculated from the 6.22 mM^−1^ cm^−1^ extinction coefficient. GST enzyme activity was calculated by measuring the conjugation of GSH with excess 1-chloro-2,4-dinitrobenzene (CDNB) at A_340_ as described by Habig et al. [62]. The NBT assay was carried out to determine the xanthine oxidase (XO) activity by following the methodology of Ozer et al. [63], and the absorbance was recorded at 575 nm. The soluble protein content was estimated according to Lowry et al. [64].

### Determination of reduced glutathione (GSH) and reduced ascorbate (ASC) content

High-performance liquid chromatography with electrochemical detection was applied for simultaneous determination of ASC and GSH by a Reversed-Phase HPLC of Shimadzu (Hai Zhonglu, Shanghai). Tissues were homogenized using a mortar and pestle under liquid nitrogen. The resulting powder was thawed on ice in a 6% metaphosphoric acid (MPA) solution (0.5 ml MPA/100 mg wet tissue). After homogenization, the samples were centrifuged at 14,000 rpm for 12 min. 100 µL of the supernatant was added to 300 µL eluens (2 mM KCl, adjusted to pH 2.5 with ortho phosphoric acid). Anti-oxidants were separated on HPLC by injecting 10 µL onto a Polaris C18-A column (3 µm particle diameter, 100 mm, 4.6 internal diameter, Varian) with a 1 mL/min flow rate (Shimadzu autoinjector SIL-10ADVP, Shimadzu isocratic pump LC 10-ADVP, 90 bar pressure, Shimadzu degasser DGU-14A). The different components were identified and quantified using an amperometric detection system (glassy carbon working electrode, calomel reference electrode, reference potential 500 mV) in series with a diode array detector (SPDM10AVP, Shimadzu,'s Hertogenbosch, Netherlands). Chromatogram analysis was performed with the ClassVP software package from Shimadzu.

The concentrations of reduced glutathione (GSH), total glutathione (tGSH), reduced ascorbate (ASC) and total ascorbate (tASC) were calculated using a standard curve created by known concentrations of GSH and ASC and expressed in terms of nmol/g wet weight. The standards were prepared freshly before use (Peak ASC: 242 nm, peak GSH: 196 nm; Retention time of ASC was 1.7–1.8 min and of GSH 2.2–2.3 min). Oxidized glutathione (GSSH) content was calculated as the difference between the content of tGSH and GSH. Similarly, the content of oxidized ascorbate (dehydroascorbate, DHA) represents the difference between tASC and ASC.

### Statistical analysis

All data have been presented as mean values ± standard error (S.E.). Within species, no significant differences were found between any of the control values at different sampling times. Therefore, pooled controls for each experimental group were used. For comparisons between different experimental groups a one-way analysis of variance (ANOVA) was performed followed by the least significant difference (LSD) test. Student's unpaired two-tailed t-test was used for single comparisons. Pearson correlation was performed to show the relationship among various variables. The data were analyzed by Statistical Package for the Social Sciences (SPSS) version 20.0. A probability level of 0.05 was used for rejection of the null hypothesis.

## Results

### Ammonia accumulation

Exposure to 1 mM HEA resulted in an increase in ammonia concentration in the liver of all three species studied (Fig. 1A). Accumulation was significant in trout after 24 h exposure and persisted until the end of the exposure period (180 h). It followed the same pattern in carp and goldfish, but in these fish the increase was delayed and became significant (*P*<0.05) from 48 h onwards. Little change (*P*>0.05) was observed in gill tissue in all three fish species (Fig. 1B).

**Figure 1:** Ammonia accumulation. Ammonia accumulation (µmol/g) in (A) liver and (B) gills of rainbow trout, common carp and goldfish during 1 mM ammonia exposure. Values are mean ± S.E. Asterisk (*) indicates a significant difference between the exposed fish and its respective control (*P<0.05).

No mortality was noted for any of the fish species during the whole experimental period.

### Oxidative stress indicators

#### H_2_O_2_ content

HEA induced a production of H_2_O_2_ in the liver in all three fish species (Fig. 2A). The effect was more prominent in trout; the level increased (*P*<0.05) from 24 h onwards. In carp, a transient increase (50% and 39% at 24 h and 48 h respectively, *P*<0.05) was followed by a recovery thereafter. Also in goldfish, a transient rise was seen at 48 h HEA (49% increment; *P*<0.05). In branchial tissue, only trout showed a significant rise during the last two exposure times (49% and 47% at 84 and 168 h HEA respectively, *P*<0.05, Fig. 2B).

**Figure 2:** Hydrogen peroxide content. Hydrogen peroxide (H_2_O_2_) content (nmol/g) in (A) liver and (B) gills of rainbow trout, common carp and goldfish during 1 mM ammonia exposure. Values are mean ± S.E. Asterisk (*) indicates a significant difference between the exposed fish and its respective control (*P<0.05; **P<0.01).

#### MDA content

Liver lipid peroxide (MDA) content displayed the same pattern as H_2_O_2_ production in all three species. In trout, a significant rise (∼52% and 58% increment at 24 h and 48 h respectively; *P*<0.05) reduced slightly but remained significantly higher than the control (Fig. 3A). In comparison to control, carp displayed a relative increment of 44% and 49% (*P*<0.05) at 24 h and 48 h exposure respectively. MDA content increased by 40% (*P*<0.05) in 48 h exposed goldfish. Such augmentations were delayed and less prominent in gill tissue. A significant increment of ∼43% occurred in trout gills from 48 h onwards (*P*<0.05; Fig. 3B). Elevations of MDA in carp and goldfish were only detected at 84 h exposure and were 55% and 47% (*P*<0.05) higher than their respective controls.

**Figure 3:** Malondialdehyde content. Malondialdehyde (MDA) content (nmol/g) in (A) liver and (B) gills of rainbow trout, common carp and goldfish during 1 mM ammonia exposure. Values are mean ± S.E. Asterisk (*) indicates a significant difference between the exposed fish and its respective control (*P<0.05).

#### Xanthine oxidase (XO) activity

XO activity in liver increased in response to HEA in all three fish species, and increments in trout were again more pronounced (Fig. 4A). Activity enhanced by 39% (*P*<0.05), 43% (*P*<0.05), 74% (*P*<0.01) and 70% (*P*<0.05) respectively after 24 h, 48 h, 84 h and 180 h. The induction was postponed in carp and goldfish, and an increment was prominent from 48 h and 84 h onwards respectively. The relative increase (*P*<0.05) in carp liver was 46%, 50% and 60% after 48 h, 84 h and 180 h respectively while goldfish showed 41% and 40% increment (*P*<0.05) after 84 h and 180 h. In contrast, HEA exerted a mild effect in gills; trout XO activity was significantly increased after 180 h exposure (Fig. 4B), carp and goldfish showed no significant trend.

**Figure 4:** Xanthine oxidase activity. Xanthine oxidase (XO) activity (nmol/min/mg protein) in (A) liver and (B) gills of rainbow trout, common carp and goldfish during 1 mM ammonia exposure. Values are mean ± S.E. Asterisk (*) indicates a significant difference between the exposed fish and its respective control (*P<0.05; **P<0.01).

### Antioxidant enzyme activities

In both goldfish and carp, SOD activity increased (*P*<0.05), respectively from 24 h and 48 h up to 84 h (Fig. 5A). These increases were followed by a partial recovery at the last exposure period. However, such an increment was delayed in trout and became significant only after 180 h of exposure. The activity remained unchanged in gills of both salmonid and cyprinids when subjected to HEA (Fig. 5B).

**Figure 5:** Superoxide dismutase activity. Superoxide dismutase (SOD) activity (units SOD/mg protein) in (A) liver and (B) gills of rainbow trout, common carp and goldfish during 1 mM ammonia exposure. Values are mean ± S.E. Asterisk (*) indicates a significant difference between the exposed fish and its respective control (*P<0.05; **P<0.01).

Ammonia exposure induced differential changes in CAT activity among cyprinid and trout liver (Fig. 6A). Our results showed that CAT activity in liver of goldfish and carp elevated respectively from 48 h and 84 h onwards (*P*<0.05). The relative increment (*P*<0.05) in goldfish was 52%, 47% and 50% after 48 h, 84 h and 180 h respectively, while in carp the average elevation (during 84 h–180 h) was 47% compared to its control value. In contrast, CAT activity did not increase (*P*>0.05) in trout on HEA exposure. Similar to SOD, branchial CAT activity remained unaltered throughout the 180 h exposure period in all the three experimental fish species (Fig. 6B).

**Figure 6:** Catalase activity. Catalase (CAT) activity (µmol H_2_O_2_/min/mg protein) in (A) liver and (B) gills of rainbow trout, common carp and goldfish during 1 mM ammonia exposure. Values are mean ± S.E. Asterisk (*) indicates a significant difference between the exposed fish and its respective control (*P<0.05).

The activity of APX in liver of carp increased gradually in response to HEA exposure and became significant after 24 h (28% increment; *P*<0.05), reached a peak at 48 h (42% increment; *P*<0.05), and declined slightly thereafter but remained significantly higher than control levels (Fig. 7A). Such an induction was somewhat delayed in gills where an effect was noted from 84 h onwards (Fig. 7B). A distinct increased (*P*<0.05) APX activity in liver and gills of goldfish was also detected after 48 h and 180 h exposure respectively while liver and gills of trout did not appear to be affected by HEA.

**Figure 7:** Ascorbate peroxidase acivity. Ascorbate peroxidase (APX) acivity (µmol ASC/min/mg protein) in (A) liver and (B) gills of rainbow trout, common carp and goldfish during 1 mM ammonia exposure. Values are mean ± S.E. Asterisk (*) indicates a significant difference between the exposed fish and its respective control (*P<0.05).

Though no stimulation of CAT and APX activity was noted for HEA exposed trout, significant (*P*<0.05) 49%, 46% and 50% increases in hepatic GR activity were observed for this species after 48 h, 84 h and 180 h of HEA exposure (Fig. 8A) and in gill after 84 h of HEA (Fig. 8B). In contrast, no significant increases in hepatic or branchial GR activity were observed in goldfish or carp.

**Figure 8:** Glutathione reductase activity. Glutathione reductase (GR) activity (nmol NADPH/min/mg protein) in (A) liver and (B) gills of rainbow trout, common carp and goldfish during 1 mM ammonia exposure. Values are mean ± S.E. Asterisk (*) indicates a significant difference between the exposed fish and its respective control (*P<0.05).

Species-wise response of hepatic GPX activities showed a significant increment in trout (during 48–180 h) and goldfish (during 84 h) only (Fig. 9A). No alteration was seen for branchial GPX activity for any of the three fish species (Fig. 9B). Regardless of exposure time, species or organ, HEA did not induce notable change in GST activity (data not shown).

**Figure 9:** Glutathione peroxidise activity. Glutathione peroxidise (GPX) activity (nmol NADPH/min/mg protein) in (A) liver and (B) gills of rainbow trout, common carp and goldfish during 1 mM ammonia exposure. Values are mean ± S.E. Asterisk (*) indicates a significant difference between the exposed fish and its respective control (*P<0.05).

### Antioxidant molecules

#### Reduced ascorbate (ASC) and ASC to DHA ratio

Exposure of cyprinids to HEA induced an increase of [ASC] in both liver and gills while no significant change occurred in exposed trout (Fig. 10A, 10B). In carp liver, this increase was notable from 24 h onwards (*P*<0.05), with a transient reduction at 48 h (Fig. 10A). In goldfish, a relative increase of 26% (*P*<0.01) and 22% (*P*<0.01) was observed after 84 h and 180 h respectively. The ratio of ASC to DHA in liver of all three fish species revealed almost the same pattern as seen for [ASC] (Table 1). In carp, this ratio increased after 48 h, 84 h and 180 h by 25% (*P*<0.05), 32% (*P*<0.001) and 29% fold (*P*<0.01) respectively. Likewise, a relative rise of 21% (*P*<0.05) and 23% (*P*<0.05) was evident in goldfish during 84 h and 180 h. The rise in [ASC] and ASC/DHA was delayed in gills of cyprinids; carp exhibited a significant augmentation only during the last two exposure phases. It was further postponed in goldfish where an elevation was noted only during the last exposure period (Fig.10B, Table 1).

**Figure 10:** Reduced ascorbate (ASC) content. Concentration (nmol/g) of reduced ascorbate (ASC) in (A) liver and (B) gills of rainbow trout, common carp and goldfish during 1 mM ammonia exposure. Values are mean ± S.E. Asterisk (*) indicates a significant difference between the exposed fish and its respective control (*P<0.05; **P<0.01).

**Table 1:** Ascorbate (ASC)/Dehydroascorbate (DHA) ratio and glutathione (GSH)/oxidized glutathione (GSSH) ratio in liver and gills of rainbow trout, common carp and goldfish during 1 mM ammonia exposure.

		Control	3 h	12 h	24 h	48 h	84 h	180 h
**[ASC]/[DHA]**								
Liver	Rainbow trout	6.51±0.45	6.08±0.67	5.67±0.61	5.82±0.56	6.24±0.72	7.07±0.46	6.85±0.59
	Common carp	7.42±0.61	7.31±0.45	7.78±1.08	8.75±0.76	9.28±0.54^*^	9.76±0.67^***^	9.54±0.51^**^
	Goldfish	7.26±0.60	6.87±0.52	7.33±0.65	7.86±0.76	7.76±0.77	8.77±0.61^*^	8.91±0.58^*^
Gills	Rainbow trout	6.08±0.45	5.66±0.43	5.89±1.09	6.17±0.76	6.78±1.08	5.98±0.87	6.18±0.55
	Common carp	7.12±0.56	7.45±0.78	6.78±1.08	7.06±0.71	7.98±0.52	8.69±0.61^**^	8.56±0.62^*^
	Goldfish	7.21±0.52	7.11±0.78	6.79±0.34	6.43±0.61	7.19±0.70	7.86±0.68	8.87±0.62^*^
**[GSH]/[GSSH]**								
Liver	Rainbow trout	7.22±0.57	6.85±0.72	7.06±1.07	7.30±0.88	8.45±0.76	9.61±0.71^*^	9.22±0.61^*^
	Common carp	6.61±0.65	6.75±0.43	6.35±0.55	5.97±0.91	6.89±0.46	7.56±0.67	7.43±0.71
	Goldfish	6.88±0.52	7.15±0.56	6.44±0.78	7.78±0.81	7.75±0.67	8.89±0.86^*^	9.05±0.91^*^
Gills	Rainbow trout	6.75±0.67	5.56±0.45	5.67±0.87	6.89±1.22	6.17±0.70	7.18±0.73	8.59±0.74^*^
	Common carp	6.32±0.45	6.67±1.21	5.67±0.86	5.78±0.78	7.12±0.51	6.78±0.62	7.25±0.66
	Goldfish	6.46±0.52	5.67±0.67	5.88±0.97	6.06±1.08	7.67±0.64	7.12±0.45	8.06±0.62^*^

Values are mean ± S.E. Asterisk (*) indicates a significant difference between the exposed fish and its respective control (*P<0.05;**P<0.01;***P<0.001).

#### Reduced glutathione (GSH) and GSH to GSSH ratio

A significant induction in [GSH] was noted in liver and gill of trout in response to HEA (Fig.11A, 11B). In liver, [GSH] increased significantly from 48 h onwards while in gill an elevation was noted at 180 h exposure (*P*<0.05). No increase or decrease occurred in liver and gills of carp. However, goldfish liver responded with a 26% (*P*<0.05) and 24% (*P*<0.05) increment after 84 h and 180 h of HEA exposure respectively. There was no alteration in gill tissue. Basal [GSH] in trout liver was approximately 1.6 times higher (*P*<0.001) than in carp and goldfish. Also in gills tissue, trout possessed 1.8 times higher (*P*<0.001) level of basal GSH content than cyprinids.

**Figure 11:** Reduced glutathione (GSH) content. Concentration (nmol/g) of reduced glutathione (GSH) in (A) liver and (B) gills of rainbow trout, common carp and goldfish during 1 mM ammonia exposure. Values are mean ± S.E. Asterisk (*) indicates a significant difference between the exposed fish and its respective control (*P<0.05).

Trout liver displayed a relative increase of 33% (*P*<0.05) in the GSH/GSSH ratio from 84 h onward, and a similar rise of 30% (*P*<0.05) was observed in goldfish (Table 1). In contrast to trout and goldfish, exposure to HEA did not induce noteworthy changes in carp although the value tended to increase with exposure period. Branchial tissue of trout and goldfish followed the same pattern for GSH/GSSH ratio, with a significant effect during the last exposure period.

Pearson correlation among the various variables in the liver of trout, carp and goldfish is illustrated in Table 2. No significant correlations were found in gill tissue.

**Table 2:** Correlations among various variables investigated in the liver of rainbow trout, common carp and goldfish during 1

	Ammonia content	H_2_O_2_	MDA	XO	SOD	CAT	ASC	APX	GSH	GPX	GR
**Rainbow trout**											
H_2_O_2_	0.342*										
MDA	0.240	0.396**									
XO	0.332*	0.219	0.314*								
SOD	0.216	0.245	0.155	0.179							
CAT	−0.006	0.017	0.083	0.107	0.276*						
ASC	0.049	0.073	0.080	0.219	0.184	0.116					
APX	0.202	−0.076	−0.096	0.027	0.175	−0.193	−0.179				
GSH	0.371**	0.332*	0.204	0.459**	0.249	0.184	0.135	−0.064			
GPX	0.004	0.345*	0.071	0.294*	0.229	0.396**	0.142	−0.010	0.280		
GR	0.274	0.450**	0.370**	0.218	0.241	0.177	0.180	0.067	0.404**	0.224	
GST	−0.101	−0.170	−0.190	−0.176	0.075	0.241	0.019	0.037	0.185	−0.022	0.060
**Common carp**											
H_2_O_2_	0.323*										
MDA	0.141	0.163									
XO	0.306*	0.066	0.011								
SOD	0.124	0.174	0.159	0.445**							
CAT	0.283*	−0.059	0.122	0.167	0.147						
ASC	0.025	0.092	0.118	0.098	0.088	0.132					
APX	0.016	−0.001	0.306*	0.374**	0.102	0.309*	0.329*				
GSH	0.051	0.023	0.232	0.025	0.140	−0.123	0.234	0.152			
GPX	0.153	0.139	0.109	0.115	0.226	−0.029	0.143	0.050	0.275*		
GR	0.255	0.326*	0.220	0.109	0.217	0.348*	−0.127	0.108	0.116	0.157	
GST	0.323*	0.088	0.051	0.050	0.132	0.198	0.265	0.112	0.203	0.108	0.084
**Goldfish**											
H_2_O_2_	0.431**										
MDA	0.358*	0.106									
XO	0.511**	0.409**	−0.025								
SOD	0.396**	0.451**	0.032	0.387**							
CAT	0.193	0.135	0.182	0.114	0.168						
ASC	0.124	0.011	−0.075	0.243	0.055	0.325*					
APX	0.242	−0.024	0.206	0.009	0.218	0.348*	0.442**				
GSH	0.130	0.093	0.359*	0.138	0.040	0.179	0.271	0.236			
GPX	−0.053	0.052	0.160	−0.115	0.107	0.214	0.154	0.283*	0.255		
GR	0.138	0.110	0.041	0.071	0.066	0.081	0.233	0.199	0.192	0.316*	
GST	0.243	−0.118	0.165	0.141	0.213	0.214	0.129	0.223	0.166	−0.002	0.070

The listed values are the correlation coefficient (r).

*Correlation is significant at 0.05 level (2-tailed).

**Correlation is significant at 0.01 level (2-tailed).

## Discussion

### Ammonia- mediated oxidative stress

A high level of ammonia in aquatic environments is toxic for many reasons, one of which is that ammonia can induce oxidative stress in fish [30]–[32], [65]. In the present study, exposure to 1 mM ammonia led to a substantial increase in ammonia content in the liver of both trout and cyprinids and was accompanied by a differential oxidative stress response. We examined the level of H_2_O_2_ and MDA production along with the activity of XO, as biomarkers of oxidative stress. The production rate of H_2_O_2_ in the liver of all the fish species elevated in response to HEA but was restored to control level only in carp and goldfish. H_2_O_2_ content was positively (*P*<0.05–0.01) correlated with ammonia accumulation in the hepatic cells of all the three fish species (Table 2). In general, excess H_2_O_2_ (and O_2_^• −^) can be transformed (via the Haber–Weiss reaction) to form highly reactive oxidant hydroxyl radicals (^•^OH) that lead to lipid peroxidation through degradation of polyunsaturated fatty acids (PUFAs). Malondialdehyde (MDA), the oxidative end product of PUFAs increased in both trout and cyprinid liver under ammonia stress. Increases in lipid peroxidation in response to ammonia exposure have been reported for Nile tilapia [31], [66], mudskipper (*Boleophthalmus boddarti*) [30], bighead carp (*Hypophthalmythys nobilis*) [32] and silver carp (*Hypophthalmichthys molitrix*) [65]. Furthermore, similar to the H_2_O_2_ response, elevated MDA levels in trout persisted longer and failed to re-establish to control levels in contrast to MDA levels in cyprinids. It is very likely that during ammonia stress, carp and goldfish could effectively remove ROS including H_2_O_2_ from early stage of lipid peroxidation limiting the accumulation of terminal products of lipid peroxidation (MDA). These alleviated lipid peroxidation in cyprinids might be due to a more efficient anti-oxidative defence (discussed below) compared to trout. Additionally, the most common PUFA present in fish species is eicosapentanoic acid (EPA) which is highly susceptible to lipid peroxidation [67], [68]. Salmonid tissues are characterized by the presence of high concentrations of PUFA in general, and EPA in particular, compared with most fish and mammalian tissues [69], [70]. Therefore, salmonids are prone to lipid per-oxidative cellular injury [45]. This could explain in part the occurrence of more prolonged and intense ammonia mediated oxidative stress in trout in contrast to cyprinids. This is also apparent by the significant positive correlation (r = 0.396, *P*<0.01) between H_2_O_2_ level and MDA content in trout.

In general, oxidative metabolism of cells is a continuous source of ROS, and in biological systems about 10% of consumed oxygen is transformed via one-electron reductions to ROS [41]. In this context, biological activity such as fast swimming or severe exercise which increases oxygen intake and metabolism, particularly in hepatic tissue and skeletal muscle, has long been postulated to cause oxidative stress and associated tissue damage [71], [72] which was confirmed by Aniagu et al. [73] in adult chub (*Leuciscus cephalus*). High-performance swimmers like salmonids used in the present study perpetually exercise, consequently ROS production rate in these fish are possibly higher than in average swimmers like cyprinids.

However, the mechanisms by which ammonia induces free radical production and oxidative stress is poorly understood in fish. In brain tissue of mammals the high accumulation of glutamine as a result of the ammonia intoxication process, is suggested to induce oxidative stress [17], [74]. Elevation in glutamine level can cause astrocyte swelling, and/or activation of *N*-methyl-D-aspartate type glutamate (NMDA) receptors [75]–[78]. The over-activation of NMDA receptors incites excess production of ROS and reactive nitrogen species [79]. For the piscine group, some evidence favour over-activation of the glutamate NMDA receptors as the consequence of ammonia toxicity [80], [81], while recent research suggest that HEA can even cause oxidative damage in gills, liver and muscle that lacks NMDA receptors [30]–[32], [38]. Apparently, there are other routes by which HEA can induce oxidative stress in fish liver and gills. Nevertheless, ROS are also produced by a cascade of oxidative enzymes such as XO, aldehyde oxidase (AOX), hydroperoxidase (HPX) and other peroxisomal enzymes [82], [83]. Among these, XO uses molecular oxygen as the electron acceptor and releases substantial amounts of O_2_^• −^ and H_2_O_2_. The species-wise response of XO activity in liver revealed a positive correlation (*P*<0.05–0.01) with ammonia accumulation, reinforcing that elevated internal ammonia levels may be involved in the signalling mechanism for the up-regulation of this enzyme and thereby for the free radical production. Likewise, in ammonia-exposed Nile tilapia the activity of XO in liver and muscle was significantly elevated; confirming this activation as the vital factor for the increased rate of ROS production under ammonia threat [31]. Trout displayed a much earlier and enhanced response of hepatic XO activity compared to carp and goldfish. This might be another justification for persistent occurrence of significant higher H_2_O_2_ and MDA content in trout compared to cyprinids. Nevertheless, as a limitation of this analysis we need to acknowledge that the activity of other enzymes contributing to the cellular redox status (e.g. AOX, HPX), were not measured.

In general, ammonia is considered as potent neurotoxin that predominantly affects the brain tissue. Besides causing astrocyte swelling, interfering with amino acid transport as well as excitatory amino acid neurotransmitter metabolism; ammonia neurotoxicity also appears to induce oxidative stress. In our previous same comparative study [84] we reported the conversion of accumulated ammonia to glutamine and other free amino acids as a potential mechanism to avoid ammonia toxicity in brain tissue. In addition, brain tissues contain high levels of lipids, which are particular prone to oxidation. Consequently, the investigation of oxidant/antioxidant systems in brain tissue would offer a better understanding to link between ammonia exposure, glutamine accumulation and induction of oxidants. However, the constraint of this study need to be mentioned, due to lack of brain samples the oxidative and anti-oxidative status in this nervous system were not investigated.

### Ammonia induced anti-oxidant defence mechanism

#### ROS scavenging enzymes - SOD, CAT and APX

A weak response of SOD in trout liver suggests that unlike cyprinids, it does not seem to rely on SOD as their first defence to counter ammonia-mediated ROS production. Similarly, when confronted with water-borne copper a very limited activation of SOD was noted for rainbow trout in comparison to common carp and gibel carp (*Carassius auratus gibelio*) [46]. SOD appears to be the key enzyme that catalyses H_2_O_2_ synthesis. Surprisingly, in trout H_2_O_2_ content was elevated considerably during HEA (24 h–180 h) despite the fact that SOD activities were not activated significantly, though an increasing trend of SOD activity was observed in response to HEA. It is possible that the higher resting SOD activity in trout provided more than enough H_2_O_2_ synthetic capacity and apparently it is not the only effective mechanism (at least in trout) to regulate H_2_O_2_ production. Reports on XO-derived ROS production frequently address XO as the O_2_^• −^ producers and H_2_O_2_ as a secondary by-product of spontaneous or enzymatic dismutation of O_2_^• −^. However, a recent study confirmed H_2_O_2_ as the dominant (70–95%) reactive product catalyzed by XO [40] favouring that during ammonia threat, H_2_O_2_ production, particularly in trout, is preferably regulated by XO since H_2_O_2_ production was accompanied by a parallel increment of XO activity. In carp and goldfish, hepatic SOD activity first increased and then returned to the control level at the end, possibly suggesting some sort of recovery response or a limited production of ROS at the end of the exposure period.

CAT is one of the primary antioxidant enzymes involved in the elimination of H_2_O_2_ which is a by-product of the SOD activity. An elevated rate of CAT activity in the liver of carp and goldfish in response to ammonia might partly explain the restoration of H_2_O_2_ content to basal level. Likewise, the activity of CAT in liver of Nile tilapia and in bighead carp larvae was reported to significantly increase due to ammonia exposure [31], [32]. However, CAT activity remained statistically unaltered in trout highlighting their lower ability, relative to cyprinids, in scavenging H_2_O_2_ resulting in a consistent elevated level of H_2_O_2_ throughout the exposure period. Similar results were found in an earlier comparative study on rainbow trout and cyprinids in response to copper exposure; no change in CAT activity was noted for trout while cyprinids displayed a significant induction [46].

Besides CAT, APX is another major enzymatic cellular scavenger of H_2_O_2_ but unlike CAT, APX needs a reductant, ascorbate (ASC). The dynamics of hepatic APX in trout and cyprinids to HEA exposure was analogous to CAT, reflecting advanced capability of carp and goldfish over trout to keep a low level of H_2_O_2_ and prevent ROS from poisoning cells.

#### ASC- GSH dependent pathway

An increased ASC pool and ASC/DHA value is an indicator of the adaptive response to limit the oxidative damage in fish [46], [85]. The high levels of reduced [ASC] in response to HEA connote an advantage for the carp and goldfish to resist oxidative stress. Interestingly, the increment of APX activity was not associated by a concomitant reduction of [ASC] in both carp and goldfish suggesting an efficient replenishment of ASC consumed via APX -based H_2_O_2_ quenching, possibly through the over expression of dehydroascorbate reductase and monodehydroascorbate reductase. Both of these enzymes recycle oxidized forms of ascorbate (DHA) into ASC. Therefore, investigation of the activity of these enzymes may be crucial in future experiments.

GSH acts as a substrate or cofactor for various enzyme reactions of the glutathione-dependent cycle and is involved in the decomposition of H_2_O_2_ to water and in the reduction of lipid hydroperoxides. Thus, a change in GSH levels may be an important indicator of the defence ability of an organism against oxidative stress [86]. Rainbow trout was characterized by a high GSH content in the liver, almost 1.6 times more compared to the cyprinids. Moreover, a significant increment in trout [GSH] was seen in response to HEA, which showed a positive correlation with ammonia accumulation (r = 0.371, *P*<0.01) and H_2_O_2_ content (r = 0.332, *P*<0.05; Table 2). It is tempting to think that the elevated basal level and hyper- responsiveness of GSH in trout may be compensatory to the poor CAT, SOD and ASC system in this species. This suggests that the GSH dependent pathway might be the most preferred anti-oxidative mechanism in rainbow trout, which corroborates the findings of Hansen et al. [87] and Eyckmans et al. [46] in copper exposed trout. Similar to trout, goldfish, but not carp, also seem to rely on GSH pathway for scavenging ROS. In a recent study on bighead larvae, Sun et al. [32] also reported an increment in GSH content with increasing NH_3_–N concentrations in rearing water. Furthermore, at the expense of GSH, GPX catalyses the reduction of H_2_O_2_ and lipid peroxides but during this process GSH is oxidized to GSSH. The activity of GPX in the ammonia exposed trout and goldfish liver tissue was significantly elevated signifying a rise in [GSSH]. The metabolic equilibrium towards the synthesis of GSSH is an indication of oxidative stress. Conversely, both trout and goldfish maintain a high intracellular GSH/GSSG ratio during exposure (84 h–180 h) suggesting an efficient elimination of GSSH from the system. GR reduces the oxidized glutathione (GSSH) to GSH in a NADPH dependent pathway, and the normal implementation of this redox- cycle maintains a high intracellular GSH pool and GSH/GSSH ratio. When its activity increases, more GSSG is converted in GSH. Subsequently, parallel increments in GR activity along with GPX activity in exposed trout explain an efficient replenishment of GSH. Interestingly, our results also indicate that the liver of goldfish was able to increase glutathione production in response to HEA, and it could maintain a relatively high GSH/GSSH ratio in spite of a lack of increment in GR activity. Likewise, in ammonia polluted water an increase in [GSH] and GSH/GSSH ratio was reported in brain of mudskippers, marked by a decline in GR activity [30]. Gamma-glutamyl cysteine synthetase has also been documented for producing GSH in cells, and an increase in the activity of this enzyme was reported under acute hyperammonemic conditions [88]. Presumably, these additional routes could have contributed to the increase in GSH levels in goldfish and mudskipper exposed to ammonia. In contrast to goldfish, in carp neither the [GSH] nor the array of enzymes involved in glutathione dependent catalytic cycle was affected by HEA, illustrating a divergent pattern of anti-oxidative response even within the species of same piscine *Cyprinidae* family. GSH also serves as a cofactor for GST activity which facilitates the detoxification of xenobiotics or reactive molecules by forming conjugates with glutathione. The activity of GST remained unaltered in all the species signifying its inconsequential role in ammonia detoxification. Taken together, our results demonstrate that exposure to HEA elicits pro-oxidant conditions since it triggered adaptive responses marked by increases in the constitutive levels of antioxidant enzymes and molecules.

In the present study, feeding was suspended 2 days prior to the experimentation. However, ammonia dynamics and tolerance in fish appear to be affected by feeding. Wicks and Randall [29] reported that during ammonia exposure, feeding could greatly up-regulate glutamine synthetase activity and glutamine levels in brain and liver tissue of rainbow trout compared to the fasted group. Consequently, it is appealing to speculate that a higher, feed-activated, glutamine synthesis might manipulate anti-oxidant/pro-oxidant systems in fish under ammonia threat. This issue provides a cautionary note as to the importance of considering feeding as a crucial factor in future related studies.

### Tissue specificity of the anti-oxidant response

Tissue-specific response shows that ammonia induced only a mild oxidative stress in gills. This could be due to slower and mild ammonia accumulation in gill, but also because liver, beside plasma and brain, is the important site of multiple oxidative metabolisms, maximal free radical generation and ammonia synthesis. In our earlier comparative study [89] investigating the same level of ammonia (1 mM), ammonia excretion (via gills) was strongly stimulated in response to HEA in carp and goldfish while trout exhibited insignificant increments. These improved excretion rates might correspond to the insignificant ammonia build-up in gills in the fish in this study. It was apparent that induction of anti-oxidative responses in gill tissues of the three fish species was almost negligible, and when present, limited to the last exposure time. Comparison between hepatic and branchial tissue in the present study suggests that ammonia accumulation, and therefore ammonia mediated overproduction of ROS, is mainly a problem in liver leading to a distinctively high anti-oxidative protective response in hepatic tissue. In general, the liver is the major source of GSH levels in blood and is the main storage organ for GSH prior to exportation to other organs [44]. Accordingly, in the present study, glutathione mediated anti-oxidative responses in all the three fish species were more pronounced in liver compared to gills. Overall, our results indicate that trout, carp and goldfish have a reduced need of anti-oxidant response in gills during HEA threat.

### Time lag- response dynamics

On the basis of the analysis above, the dynamics of oxidative stress and associated defence response in liver can be divided into three phases: steady state, oxidative stress and acclimation (fig. 12). Phase I, steady state, refers to the early phase of exposure which was characterized by the equilibrium between pro-oxidant and antioxidant defence mechanisms. In trout, this phase persisted until 12 h while in cyprinids it continued until 24 h–48 h of exposure. Phase II was marked by the incidence of oxidative stress which was associated with the activation of both enzymatic and non-enzymatic antioxidants. Species specific differences were noted at this phase, in trout ROS generation was not inhibited efficiently through the antioxidant action and therefore H_2_O_2_ concentration and lipid peroxidation (measured as MDA) remained elevated until the end of the exposure. On the contrary, carp and particularly goldfish were able to control ROS generation by anti-oxidative counteracting systems. This resulted in recovery from oxidative stress which returned to control levels in the recovery or acclimation phase during the 84 h–180 h HEA exposure.

**Figure 12:** Defence responses. A simplified illustration of the differential reactive oxygen species (ROS) production and antioxidant (AO) defence responses in liver of rainbow trout, common carp and goldfish during 1 mM ammonia exposure. Phase I (P I) represents steady state; Phase II (P II) represents oxidative stress and associated defence response, and Phase III (P III) represents acclimation or recovery stage. Note the absence of P III in rainbow trout.

## Conclusion

The results of the present study suggest that exposure to 1 mM HEA can elicit pro-oxidant conditions, which induced differential oxidative stress and anti-oxidative compensatory responses among the three freshwater teleosts. The effect was more evident in the liver compared to the gills. The increase in hepatic activity of XO in all three species stimulated H_2_O_2_ production which was manifested by a rise in MDA content. To neutralize the impact of oxidative damage, both enzymatic and non-enzymatic antioxidants were activated and species-specific differences were profound. In response to HEA, SOD and CAT activity increased only in cyprinids with a very mild increment of SOD in trout. On the contrary, trout relied mainly on the components of the glutathione cycle to counteract the ROS generation as they possessed high levels of GSH and showed a significant increment in [GSH], and activity of GPX and GR. Goldfish also appear to rely on the GSH redox pathway; however, carp could not implement this pathway as an antioxidant defence. ASC levels and APX were augmented only in carp and goldfish while trout did not show any remarkable response. Therefore, it is apparent that the anti-oxidative defence system in trout is not as proficient as in carp while goldfish revealed a well developed defensive system. This species-specific variation in compensatory response further elucidate that the trout could not fully counteract the ammonia-induced ROS generation, evident by persistent elevated levels of H_2_O_2_ and MDA until the last exposure period, whereas the carp and particularly the goldfish were able to restore the stress to basal levels (84 h–180 h). Present findings suggest that goldfish have more effective anti-oxidant system in hepatic tissue to deal with ammonia exposure than do carp, while trout appear to be least effective. Consequently, improved defence mechanisms against oxidative stress may contribute in part to the high ammonia tolerance in goldfish, with a high 96 h LC_50_ ammonia value of 4.2 mM [52] compared to common carp (2.6 mM) [49] and trout (1.7 mM) [50]. Furthermore, responses were reduced in branchial tissue, correlating to the insignificant increment in ammonia accumulation in gills. Ammonia is also a potent neurotoxin, the brain being the target organ for ammonia toxicity. Therefore, future studies on anti-oxidant status in brain tissue are warranted to provide concrete evidence contributing to the ammonia tolerance capacity in fish species. Nevertheless, the possible signalling mechanisms inducing ROS production and associated lipid peroxidation during high ammonia load need to be investigated. In addition, the regulation of these anti-oxidative enzymes at the transcriptional level might be crucial in further examinations.
